The article "The Prevalence and Association of Stress Urinary Incontinence, Core Muscle Endurance, and Low Back Pain among Married Women in Saudi Arabia: A Case-Control Study" was published in 2021. Journal: Biomed Res Int.

# The Prevalence and Association of Stress Urinary Incontinence, Core Muscle Endurance, and Low Back Pain among Married Women in Saudi Arabia: A Case-Control Study

**DOI:** 10.1155/2021/5533241

**Published:** 2021-07-15

**Authors:** Ahmad H. Alghadir, Cynthia Tse, Amir Iqbal, Mariam Al-Khater, Ghadeer Al-Rasheed

**Affiliations:** Department of Rehabilitation Sciences, College of Applied Medical Sciences, King Saud University, Riyadh, Saudi Arabia

## Abstract

**Purpose:**

There may be a strong association among stress urinary incontinence (SUI), low back pain (LBP), and core muscle endurance (CME) in married women. This study is aimed at evaluating the prevalence and clinical association between SUI, CME, and LBP among married women in Saudi Arabia.

**Methods:**

The study was based on a case-control research design, conducted among 143 women with LBP (mean age, 32 ± 7.4 years) and 160 healthy women (mean age, 31.7 ± 6.7 years). SUI, CME, and functional disability were assessed using the international consultation on the Incontinence Questionnaire-Short Form (ICIQ-SF), prone plank test (PP), and Oswestry Disability Index for LBP-United Arab Emirates edition (ODI-UAE).

**Results:**

The prevalence of SUI was found to be 60% in the LBP group while 20% in the control group. CME revealed a stronger negative correlation with SUI in the LBP group (*r*_s_ = −0.75) than in the control group (*r*_s_ = −0.63).

**Conclusions:**

The prevalence of SUI was observed higher in women with LBP than healthy women. CME exhibited a stronger association with SUI than LBP among women with LBP compared to healthy women in Saudi Arabia. Therefore, the role of CME in SUI development or vice versa among married women with LBP may be subjected to further research.

## 1. Introduction

Urinary incontinence (UI) and low back pain (LBP) are significant conditions treated by physical therapists recognizing that treating one condition often bring changes to the other condition. It has been estimated that 84% of adult women will experience more disabling pain than adult men because of LBP at some stage in their lives [1]. In addition, UI due to LBP reportedly had a 78% prevalence in adult women [2]. Several systemic and mechanical disorders such as UI, respiratory disorders, gastrointestinal symptoms [3, 4], and impaired static balance ability [5] have been recognized and significantly correlated as risk factors for the development of LBP [6]. UI is a significant and common problem in women [7]. It is reported that 25-45% of women suffer from some extent of UI, although accurate estimation of prevalence has been not reported yet only because of lack of standardization between studies and a disinclination to disclose the symptoms [8].

UI is mostly classified as stress UI (SUI), urge UI (UUI), and mixed UI (MUI). SUI is characterized by the involuntary leakage of urine on effort or exertion and from increased intra-abdominal pressure created by sneezing or coughing. Urge UI represents leakage accompanied by or immediately preceded by a strong urge to urinate, while mixed UI involves both conditions [9]. SUI is the most common form of UI with a reported variability of 4–78% among women during coughing (77%), laughing (39%), exercising (30%), heavy lifting (30%), and moving to the bathroom (27%) [2, 10].

Increasing evidences support the theory that the core muscles play an important role in trunk control and the maintenance of continence [7, 11–14]. The “core” refers to a “box” or cylinder with the diaphragm as the roof, the pelvic floor and hip girdle muscles at the bottom, the abdominals in the front and side of the belly, and the paraspinal and gluteal muscles at the back [15]. The function of the core muscles as a spinal stabilizer is usually used in the assessment and treatment of LBP by physiotherapists [11]. It has been postulated that if an individual needs to be free of LBP and continent, the core muscles must be functioning optimally [16]. In addition to PFM, the core muscles including the abdominals and diaphragm may play an essential role in trunk control and the maintenance of continence [11–14].

Stability of the lumbar spine is achieved through the coordinated efforts of the core muscles. The transverse abdominis muscles provide spinal stability by increasing tension in the thoracolumbar fascia and assist the diaphragm in modulating intra-abdominal pressure (IAP) [11]. Elevated IAP thus increases spinal stiffness [17, 18]. The PFM contract with the abdominals during postural tasks to modulate IAP [7, 12, 17] as well as provide further mechanical support to the trunk by increasing sacroiliac joint stiffness [13]. Decreased PFM strength and endurance in women with incontinence may alter the impact of the PFM in postural control and may result in lumbopelvic pain [14].

Continence is controlled through intricate coordination of the core muscles surrounding the abdominal cavity. The PFM stabilizes the neck of the bladder [19] and increases intraurethral pressure to maintain continence [20]. In fact, its level of strength is a powerful predictor of SUI [21]. A study by Ferla et al. reported the link between the abdominal muscles and the PFM and stated that a strong abdominal muscle contraction elicits a strong PFM contraction, which is important for the control of continence, especially during a cough or sneeze [12]. In contrast, one study revealed that the postural perturbations increased PFM and abdominal muscle activity in women with incontinence and advised that the treatment plan for incontinence must include abdominal muscle rehabilitation [14]. The PFM also works synergistically with the diaphragm by providing a solid platform to increase the IAP [22]. One study reported the association between LBP, UI, and the muscles related to balance ability and found that the PFM dysfunction was strongly linked with both conditions including LBP and UI in women [2]. Thus, the abdominal muscles, PFM, and diaphragm all play important roles in the maintenance of continence.

The importance of core muscle endurance (CME) in the trunk and continence control has been reported in previous studies [7, 11]. Little is known about the association between LBP, SUI, and core endurance even though the interventions for both conditions include a detailed assessment of each component of the core muscles by physical therapists [23, 24]. One study reported an association between LBP and UI [2], and another study reported the association among LBP, UI, and static balance ability [6], in a mixed population of married and unmarried women [2, 6]. However, none of the studies reported the relationship between CME, SUI, and LBP specifically among married women although they are associated with an increased risk of developing persistent SUI because of the multiparity and LBP [25]. Therefore, this study is aimed at establishing the clinical association between SUI, CME, and LBP among married women in Saudi Arabia. We hypothesized that CME would be strongly correlated with SUI and LBP among married women. Our study will highlight the importance of CME in the assessment and treatment for both the conditions (LBP and SUI) in married women. The results of this study can be used to guide clinical interventions after understanding the relationship among CME, SUI, and LBP.

## 2. Material and Methods

### 2.1. Participants

A case-control research design was used to establish the association between CME, SUI, and LBP among married women with LBP in Saudi Arabia. Once ethical approval was granted for the study, a total of 344 married women (Saudi women) who visited two different multispecialty hospitals in Riyadh, Saudi Arabia, were recruited from the outpatient department (OPD) physiotherapy between October and December of the year 2019. The married women with LBP (for the LBP group) included in this study were newly diagnosed (incidental type of cases) as mechanical LBP by a consultant orthopedic surgeon and referred to OPD physiotherapy for physical therapy interventions. However, asymptomatic/healthy married women (for the control group) with a diagnosed case of SUI by the consultant gynecologist were recruited in the study through poster advertisements, newsletters, and online websites. The cases of SUI were differentiated from UUI and MUI using the International Consultation on Incontinence Questionnaire (ICIQ) which allows the assessment of the prevalence, frequency, and perceived cause of urinary incontinence and its impact on everyday life [26]. The early documentation of each subject was done by an assistant physiotherapist in the reception of the physiotherapy department for their demographic data including name, age (years), height (m), weight (kg), body mass index (kg/m [2]), and parity (i.e., number of children).

Each study subject was initially screened according to inclusion and exclusion criteria. Out of the 344 subjects, 143 (41.57%) were recruited in the LBP group and 160 (46.51%) were recruited in the control group, and 41 (11.92%) who did not complete and cooperate the prone plank tests [27] and during the clinical assessment, respectively, were excluded from the study. A total of 303 (88.08% of the total sample) subjects provided informed consent after being provided brief and clear information about the study as well as assured for the privacy of their data. All subjects voluntarily participated in this study.

The inclusion criteria for the LBP group were limited to married women, aged within 18 to 45 years, referred to the physical therapy department for the treatment of LBP of 6 to 12 months' duration that was not a result of spinal infection, fracture, inflammatory disease, or neurological impairment. However, the inclusion criteria for the control group were limited to asymptomatic/healthy married women, aged within 18 to 45 years, and a diagnosed case of SUI. The exclusion criteria for both LBP and control groups were as follows: unmarried/married women aged <18 years and with other types of cases of UI other than SUI and women with pregnancy, pudendal nerve injury, autonomic disorders, cardiopulmonary conditions, and urinary tract infections, who are not able to retain the actual test position of the prone plank tests during familiarization session, and who showed no cooperation in the screening session for the study.

### 2.2. Procedures

The outcomes in this study were SUI, CME, and functional disability related to LBP. Firstly, the International Consultation on Incontinence Questionnaire-Short Form (ICIQ-SF) and Oswestry Disability Index for LBP-United Arab Emirates edition (ODI-UAE) were used for assessing SUI and LBP, respectively [26, 28, 29]. The participants of both groups marked the questionnaires and returned them in a sealed envelope to us. Then, all participants of both groups were called to perform a prone plank test to assess their core muscle endurance. Data were collected by an assistant physical therapist who was blinded to the study outcomes to avoid researcher bias. All data were collected and sent for appropriate biostatistical analysis.

### 2.3. Outcomes

#### 2.3.1. Assessment of Functional Disability due to Low Back Pain

All participants with LBP underwent a spinal function assessment. ODI-UAE was used to assess the functional disability related to the lower back [30]. It was translated, validated, and culturally adapted from the original English version of the ODI (version 2.0), a disease-specific questionnaire that documents the functional level that might be restricted due to LBP [29]. It has 10 items scored from 0 to 100 and interpreted as a “disability percentage”; that is, the higher the score, the greater the degree of disability.

#### 2.3.2. Assessment of Stress Urinary Incontinence

The ICIQ-SF was used to assess the prevalence of SUI [26]. The ICIQ-SF is a valid tool that is adapted culturally among Arabic countries with satisfactory psychometric properties [28]. It comprises three scoring items explaining the perceived cause of UI and its impact on everyday life as well as one nonscored item regarding the frequency of UI. Based on the achieved scores, participants were classified as being negatively correlated with SUI if the score is -1 (*r* or *r*_s_ = −1.00), not correlated with SUI if the score is 0 (*r* or *r*_s_ = 0.00), and positively correlated with SUI if the score is +1 (*r* or *r*_s_ = +1.00) or above. The closer the coefficients are to +1.0 and -1.0, the greater the strength is of the relationship between the variables.

#### 2.3.3. Assessment of Core Muscle Endurance

CME was assessed using the clinical prone plank test [27]. The test begins with the subjects lying prone on both elbows directly under the shoulders and hands together. The subjects are then allowed to bridge off the ground while holding the head in the neutral position. Once the subjects retained the correct position, the assistant physiotherapist started the stopwatch, and the subjects were asked to hold the position for 60 seconds. Failure occurs when a straight back can no longer be maintained and the hips drop toward the floor or if the subjects were unable to preserve form for a period of 60 seconds. Subject performance was then coded as “able to perform the test” or “unable to perform.” Prior to the test, a familiarization session for the test was achieved through the demonstration of the test by the physiotherapist himself or herself then performed by the subjects until the actual test position was retained or the tester was satisfied with their progress after practicing enough the test position. The subjects who did not retain the actual test position or whose progress even after practicing enough in the familiarization session did not satisfy the tester were excluded from the study.

This prone plank test selectively recruits the rectus abdominis, transverse abdominis, and external obliques [31]. This has been validated by Schellenberg et al. for its usefulness as “an endurance test for the abdominal core flexors” and is highly compatible even in subjects with LBP [32].

### 2.4. Analysis

Data analysis was performed using SPSS software version 16 (IBM SPSS Statistics Inc., NYC, USA). Baseline characteristics and descriptive statistics were computed for the two groups. Differences between the two groups were assessed using an independent samples *t*-test. Association between LBP, UI, and CME was assessed by chi-squared analysis. A nonparametric correlational analysis was undertaken to compute the Spearman rank correlation coefficient (denoted as “*r*_s_”) to explore the correlation between CME and other variables of this study. The reporting of direction and magnitude (strength) of Spearman's rank correlation coefficient for the medicine field was used based on the previous studies [33, 34]. The level of significance (*α*) was set at 0.05 (i.e., *p* < 0.05).

## 3. Results

The data analysis revealed the results for all variables and their correlations among them as follows. Demographic data showed homogenous distribution as insignificant differences (*p* > 0.05) between the LBP and control groups in age (*p* = 0.612), height (*p* = 0.827), weight (*p* = 0.339), body mass index (*p* = 0.254), and parity (*p* = 0.781) as described in Table 1.

The percentage prevalence of SUI in the LBP group (60%) was greater than that in the control group (20%) as disclosed by ICIQ-SF scores. The adjusted prevalence ratios were 1.23 (95% CI, 1.02–1.64) and 1.26 (95% CI, 1.06–1.56) for the LBP and control groups, respectively. The findings for prevalence (%) of SUI demonstrated a significant correlation with both LBP (*p* < 0.05) and control (*p* < 0.05) groups as described in Table 2.

The result for Spearman's rank correlation coefficient advocated that there were poor to strong negative correlations among CME, SUI, ODI, age, and parity (i.e., number of children) for both groups.

The values of Spearman's rank correlation coefficient indicated that the CME had a very strong negative correlation with SUI in the LBP group (*r*_s_ = −0.75) with moderate negative correlation for both the control group (*r*_s_ = −0.63) and total sample (*r*_s_ = −0.68), respectively. The CME demonstrated a moderate and poor negative correlation with ODI in the LBP group (*r*_s_ = −0.54) and control group (*r*_s_ = −0.44), respectively, and a fair positive correlation in total sample (*r*_s_ = 0.50). Additionally, CME demonstrated a moderate negative correlation with age in both groups including the LBP group (*r*_s_ = −0.61) and control group (*r*_s_ = −0.51) and in the total sample (*r*_s_ = 0.52). Likewise, CME demonstrated a moderate negative correlation with parity in both groups including the LBP group (*r*_s_ = −0.69) and control group (*r*_s_ = −0.58) and in the total sample (*r*_s_ = 0.64) as described in Table 3.

## 4. Discussion

The aim of this study was to describe the role of CME in the development of SUI among married women with LBP. The results of the study showed a “moderate to high” negative correlation between CME and SUI in both LBP and control groups. The report established a fact that the role of CME was noteworthy in the development of SUI among married women with LBP (duration of chronicity within 6-12 months) than healthy married women. It can be explained that the weaker the endurance of the core muscles, the stronger the UI severity, the higher the perceived level of disability related to LBP, and the stronger its impact on quality of life. Therefore, our result is in line with a theory explaining that the contribution of the core muscles to trunk control and the maintenance of continence may be a common risk factor for the development of SUI and LBP in married women [25].

We found that 60% of cases with LBP exhibited SUI, a rate that is significantly higher than the 20% of cases exhibiting SUI by healthy women in the control group. This finding is in accordance with another study that reported that 78% of cases with LBP had all types of UI [2]. Moreover, Kim et al. found that the higher the UI severity, the higher the perceived level of disability due to LBP [6]. This provides further evidence that LBP is correlated with SUI; thus, the presence of UI is significantly related to the development of LBP [3, 4].

PFM strength was found to be a strong predictor of UI [21], while the ability to interrupt urine flow was compromised in females with LBP [2]. Furthermore, one study reported that PFM dysfunction was linked to the development of UI in women, especially those with LBP [6]. The finding of this study is inferring/suggesting that the SUI in women with LBP may be associated further with the alteration in the optimal function of all muscles surrounding the entire abdominal cavity. This finding is consistent with studies that explained that increased PFM function does not necessarily result in decreased LBP [35] or continence [36].

LBP has been treated with an integrated approach including exercises aimed at the diaphragm, core muscles, and PFM. Training these mentioned muscles in women with mixed UI and SUI leads to an improved/cure rate of 96% [37]. Overall, these findings explain that while PFM is important in both LBP and SUI, its function is part of a coordinated effort shared by all core muscles. A possible mechanism was suggested by Smith et al., who studied the correlation between women with and without SUI and balance and found that trunk muscle (core muscles) and PFM activities increased in women with UI, which could decrease the contribution of the muscles to postural control and result in the development of LBP [4, 5].

To our knowledge, no studies to date have examined the correlation among CME, parity, and age. In this study, the authors found a moderate correlation between CME and both parity and age. The findings of this study are consistent with the previous studies that reported that the women of all age groups (20-80 years) with UI problems were found to be significantly associated with the development of LBP, increased functional disability, and decreased balance ability than healthy women [3–6, 25]. In contrast, there was no correlation between prone bridging endurance time and age found as reported by Schellenberg et al. [32]. Age-related changes in PFM results in decreased urethral closure pressure [38], while histomorphological changes occur possibly due to mechanical stress of the levator ani muscle [39]. In contrast to the other core muscles, one study found that pathological changes of the internal fibers of the back muscles occur with increasing age [40]. Furthermore, the few studies that have examined the correlations among age, LBP, and UI were contradictory [4, 10, 41]. Some reported no significant differences, while the rest reported that age was associated with a higher risk of SUI [10] and LBP [41]. In this context, our results advocated that CME could be affected by increasing age, but causation could not be tested using this research design.

We found that reduced CME was moderately associated with increased parity. PFM strength can be influenced by parity [42]. Vaginal delivery has been established as a common cause of SUI [42, 43]. Labor and vaginal delivery may cause structural problems with the pelvic floor, pelvic organs, and PFM and damage the nerve supply [24]. Back pain was perceived more frequently in parous than nulliparous younger women [32]. Increasing parity was recognized as a risk factor for the development of LBP, although the causative factor could be the general increase of mechanical activities such as lifting and bending from childrearing instead of childbearing [44]. Our results advised that, although aging and parity are associated with decreased CME, there are conflicting data to support these variables as risk factors for LBP or SUI.

### 4.1. Limitations

There were some limitations to this study. In particular, a uniform definition of LBP is lacking. Structures in the low back share segmental innervation with urogenital structures [24]. Thus, it is conceivable that our data may reflect a doubling up effect since patients with pelvic pain may attribute it to LBP. The ODI, ICIQ-SF, and prone bridge tests are clinical rather than quantitative measures. Psychosocial and cultural factors may have also influenced the outcome readings and findings. We used the prone plank test because it is a good measure of endurance rather than strength since it requires lower levels of maximum voluntary contraction [31]. Low to moderate activation levels have been shown to sufficiently stabilize the spine [32]. Bridging endurance times were significantly shorter among patients with LBP [32]. The results of this study can be used to guide clinical interventions.

## 5. Conclusion

Our study concluded that the prevalence of SUI was observed higher in married women with LBP than without LBP, which indicated an established link among SUI, LBP, and CME. In addition, the CME unveiled a very strong and negative association with the SUI among married women with LBP than without LBP. It implies that “as the CME decreases, the chances to develop SUI increase and vice versa.” Since, physical therapists have long since recognized the association of these two conditions (LBP and SUI). Hence, getting relief in either condition of SUI and LBP by treating one often affects the other. Our study highlights the importance of CME in the assessment and treatment for both the conditions (LBP and SUI) in married women.

CME might be considered a noteworthy risk factor for the development of SUI or vice versa in married women with LBP which may be subjected to research further. Therefore, future studies could be focused on core muscle strength and endurance using quantitative measures to understand the underlying cause of LBP and SUI as well as constitute a defined effective core muscle strength training program for this subgroup to discover an improvement in their symptoms.

## Figures and Tables

**Table 1:** Sociodemographic details of the subjects (mean ± SD).

Variable	LBP group (*n* = 143)	Control group (*n* = 160)	*p* value
Age (year)	32.3 ± 7.4	31.7 ± 6.7	0.612
Height (m)	1.63 ± 0.05	1.64 ± 0.06	0.827
Weight (kg)	70.3 ± 5.6	68.9 ± 5.9	0.339
BMI (kg/m^2^)	28.4 ± 4.9	26.9 ± 6.3	0.254
Parity/no. of children	2.37 ± 1.51	2.29 ± 0.76	0.781

**Table 2:** Prevalence (%) of SUI in both LBP and control groups.

Groups	Prevalence of SUI (%)	Adjusted prevalence ratio (95% CI)	*p* value
LBP group (*n* = 143)	60%	1.23 (1.02-1.64)	0.037
Control group (*n* = 160)	20%	1.26 (1.06-1.56)	0.025

**Table 3:** Association between CME (PPT), SUI (ICIQ-SF), LBP (ODI), age, and parity (Spearman's rank correlation coefficient (*r*_s_)).

Variables (risk factors)	Total sample (*r*_s_)	LBP group (*r*_s_)	Control group (*r*_s_)
Core muscle endurance & SUI	-0.68	-0.75	-0.63
Core muscle endurance & ODI	-0.50	-0.54	-0.44
Core muscle endurance & age	-0.52	-0.61	-0.51
Core muscle endurance & parity	-0.64	-0.69	-0.58

## Data Availability

Dataset supporting the conclusions of this article is available through the corresponding author upon reasonable request.

## Abbreviations

SUI: Stress urinary incontinence
LBP: Low back pain
CME: Core muscle endurance
ICIQ-SF: International Consultation on Incontinence Questionnaire-Short Form
PPT: Prone plank test
UI: Urinary incontinence
UUI: Urge urinary incontinence
MUI: Mixed urinary incontinence
ODI: Oswestry Disability Index
*r*_s_: Spearman's correlation coefficient
PFM: Pelvic floor muscle.

## References

[1] Wáng Y. X. J., Wáng J.-Q., Káplár Z. (2016). Increased low back pain prevalence in females than in males after menopause age: evidences based on synthetic literature review. *Quantitative Imaging in Medicine and Surgery*.

[2] Bush H. M., Pagorek S., Kuperstein J., Guo J., Ballert K. N., Crofford L. J. (2013). The association of chronic back pain and stress urinary incontinence: a cross-sectional study. *Journal of Women's Health Physical Therapy*.

[3] Smith M. D., Russell A., Hodges P. W. (2014). The relationship between incontinence, breathing disorders, gastrointestinal symptoms, and back pain in women: a longitudinal cohort study. *The Clinical Journal of Pain*.

[4] Smith M. D., Russell A., Hodges P. W. (2009). Do incontinence, breathing difficulties, and gastrointestinal symptoms increase the risk of future back pain?. *The Journal of Pain*.

[5] Smith M. D., Coppieters M. W., Hodges P. W. (2008). Is balance different in women with and without stress urinary incontinence?. *Neurourology and Urodynamics*.

[6] Kim J. S., Kim S. Y., Oh D. W., Choi J. D. (2010). Correlation between the severity of female urinary incontinence and concomitant morbidities: a multi-center cross-sectional clinical study. *International Neurourology Journal*.

[7] Reynolds W. S., Dmochowski R. R., Penson D. F. (2011). Epidemiology of stress urinary incontinence in women. *Current Urology Reports*.

[8] Buckley B. S., Lapitan M. C. M. (2010). Prevalence of urinary incontinence in men, women, and children—current evidence: findings of the Fourth International Consultation on Incontinence. *Urology*.

[9] Abrams P., Cardozo L., Fall M. (2003). The standardisation of terminology in lower urinary tract function: report from the standardisation sub-committee of the International Continence Society. *Urology*.

[10] Seshan V., AlKhasawneh E., Al Hashmi I. H. (2016). Risk factors of urinary incontinence in women: a literature review. *International Journal of Urological Nursing*.

[11] Chang W.-D., Lin H.-Y., Lai P.-T. (2015). Core strength training for patients with chronic low back pain. *Journal of Physical Therapy Science*.

[12] Ferla L., Darski C., Paiva L. L., Sbruzzi G., Vieira A. (2016). Synergism between abdominal and pelvic floor muscles in healthy women: a systematic review of observational studies. *Fisioterapia em Movimento*.

[13] Pool-Goudzwaard A., van Dijke G. H., van Gurp M., Mulder P., Snijders C., Stoeckart R. (2004). Contribution of pelvic floor muscles to stiffness of the pelvic ring. *Clinical Biomechanics*.

[14] Smith M. D., Coppieters M. W., Hodges P. W. (2007). Postural response of the pelvic floor and abdominal muscles in women with and without incontinence. *Neurourology and Urodynamics*.

[15] Key J. (2010). *Back Pain-a Movement Problem E-Book: A Clinical Approach Incorporating Relevant Research and Practice*.

[16] Lee D., Lee L. Stress urinary incontinence–a consequence of failed load transfer through the pelvis.

[17] Hodges P. W., Eriksson A. M., Shirley D., Gandevia S. C. (2005). Intra-abdominal pressure increases stiffness of the lumbar spine. *Journal of Biomechanics*.

[18] Key J. (2013). ‘The core’: understanding it, and retraining its dysfunction. *Journal of Bodywork and Movement Therapies*.

[19] Junginger B., Baessler K., Sapsford R., Hodges P. W. (2010). Effect of abdominal and pelvic floor tasks on muscle activity, abdominal pressure and bladder neck. *International Urogynecology Journal*.

[20] Raizada V., Mittal R. K. (2008). Pelvic floor anatomy and applied physiology. *Gastroenterology Clinics of North America*.

[21] Baracho S. M., Da Silva L. B., Baracho E., da Silva Filho A. L., Sampaio R. F., De Figueiredo E. M. (2012). Pelvic floor muscle strength predicts stress urinary incontinence in primiparous women after vaginal delivery. *International Urogynecology Journal*.

[22] Park H., Han D. (2015). The effect of the correlation between the contraction of the pelvic floor muscles and diaphragmatic motion during breathing. *Journal of Physical Therapy Science*.

[23] Ghaderi F., Oskouei A. E. (2014). Physiotherapy for women with stress urinary incontinence: a review article. *Journal of Physical Therapy Science*.

[24] Alperin M., Cook M., Tuttle L. J., Esparza M. C., Lieber R. L. (2016). Impact of vaginal parity and aging on the architectural design of pelvic floor muscles. *American Journal of Obstetrics and Gynecology*.

[25] Smith M. D., Russell A., Hodges P. W. (2008). Is there a relationship between parity, pregnancy, back pain and incontinence?. *International Urogynecology Journal*.

[26] Avery K., Donovan J., Peters T. J., Shaw C., Gotoh M., Abrams P. (2004). ICIQ: a brief and robust measure for evaluating the symptoms and impact of urinary incontinence. *Neurourology and Urodynamics*.

[27] McGill S., Belore M., Crosby I., Russell C. (2010). Clinical tools to quantify torso flexion endurance: normative data from student and firefighter populations. *Occupational Ergonomics*.

[28] Hashim H., Avery K., Mourad M., Chamssuddin A., Ghoniem G., Abrams P. (2006). The Arabic ICIQ-UI SF: an alternative language version of the English ICIQ-UI SF. *Neurourology and Urodynamics*.

[29] Fairbank J., Couper J., Davies J., O’brien J. (1980). The Oswestry low back pain disability questionnaire. *Physiotherapy*.

[30] Ramzy R. (2008). *Validation of the Arabic Version of the Oswestry Disability Index Developed in Tunisia for Low back Pain Patients in the UAE*.

[31] Ekstrom R. A., Donatelli R. A., Carp K. C. (2007). Electromyographic analysis of core trunk, hip, and thigh muscles during 9 rehabilitation exercises. *Journal of Orthopaedic & Sports Physical Therapy*.

[32] Schellenberg K. L., Lang J. M., Chan K. M., Burnham R. S. (2007). A clinical tool for office assessment of lumbar spine stabilization endurance: prone and supine bridge maneuvers. *American Journal of Physical Medicine & Rehabilitation*.

[33] Chan Y. (2003). Biostatistics 104: correlational analysis. *Singapore Medical Journal*.

[34] Akoglu H. (2018). User's guide to correlation coefficients. *Turkish Journal of Emergency Medicine*.

[35] Mohseni-Bandpei M. A., Rahmani N., Behtash H., Karimloo M. (2011). The effect of pelvic floor muscle exercise on women with chronic non-specific low back pain. *Journal of Bodywork and Movement Therapies*.

[36] Hextall A., Bidmead J., Cardozo L., Boos K., Mantle J. (1999). Assessment of pelvic floor function in women with genuine stress incontinence: a comparison between ultrasound, digital examination and perineometry. *International Urogynecology Journal*.

[37] Hung H.-C., Hsiao S.-M., Chih S.-Y., Lin H.-H., Tsauo J.-Y. (2010). An alternative intervention for urinary incontinence: retraining diaphragmatic, deep abdominal and pelvic floor muscle coordinated function. *Manual Therapy*.

[38] Murad-Regadas S. M., Regadas F. S. P., Rodrigues L. V., Furtado D. C., Gondim A. C., Dealcanfreitas Í. D. (2011). Influence of age, mode of delivery and parity on the prevalence of posterior pelvic floor dysfunctions. *Arquivos de Gastroenterologia*.

[39] Jundt K., Kiening M., Fischer P. (2005). Is the histomorphological concept of the female pelvic floor and its changes due to age and vaginal delivery correct?. *Neurourology and Urodynamics*.

[40] Shahidi B., Parra C. L., Berry D. B. (2017). Contribution of lumbar spine pathology and age to paraspinal muscle size and fatty infiltration. *Spine*.

[41] Meucci R. D., Fassa A. G., Faria N. M. X. (2015). Prevalence of chronic low back pain: systematic review. *Revista de saude publica.*.

[42] Kepenekci I., Keskinkilic B., Akinsu F. (2011). Prevalence of pelvic floor disorders in the female population and the impact of age, mode of delivery, and parity. *Diseases of the Colon & Rectum*.

[43] Memon H. U., Handa V. L. (2013). Vaginal childbirth and pelvic floor disorders. *Women’s Health*.

[44] Mannion C. A., Vinturache A. E., McDonald S. W., Tough S. C. (2015). The influence of back pain and urinary incontinence on daily tasks of mothers at 12 months postpartum. *PLoS One*.

